The article "Application of Artificial Intelligence Nuclear Medicine Automated Images Based on Deep Learning in Tumor Diagnosis" was retracted in 2023. Reasons: signs of a paper mill; suspected computer-generated content; unreliable results or conclusions; lack of ethics approval or compliance.

# Application of Artificial Intelligence Nuclear Medicine Automated Images Based on Deep Learning in Tumor Diagnosis

**DOI:** 10.1155/2022/7247549

**Published:** 2022-01-31

**Authors:** Jian Sun, Xin Yuan

**Affiliations:** ^1^Health Management Center, Second Affiliated Hospital of Dalian Medical University, Dalian 116000, China; ^2^Nuclear Medicine Department, Second Affiliated Hospital of Dalian Medical University, Dalian 116000, China

## Abstract

In order to correctly obtain normal tissues and organs and tumor lesions, the research on multimodal medical image segmentation based on deep learning fully automatic segmentation algorithm is more meaningful. This article aims to study the application of deep learning-based artificial intelligence nuclear medicine automated images in tumor diagnosis. This paper studies the methods to improve the accuracy of the segmentation algorithm from the perspective of boundary recognition and shape changeable adaptive capabilities, studies the active contour model based on boundary constraints, and proposes a superpixel boundary-aware convolution network to realize the automatic CT cutting algorithm. In this way, the tumor image can be cut more accurately. The experimental results in this paper show that the improved algorithm in this paper is more robust than the traditional CT algorithm in terms of accuracy and sensitivity, an increase of about 12%, and a slight increase in the negative prediction rate of 3%. In the comparison of cutting images of malignant tumors, the cutting effect of the algorithm in this paper is about 34% higher than that of the traditional algorithm.

## 1. Introduction

At present, cancer is becoming the leading cause of death in China, posing a serious threat to life and health. According to the latest research statistics published by He Jie and others in the world's top authoritative journal CA: A Cancer Journal for Clinicians, Tumor Hospital of the Chinese Academy of Medical Sciences, China has 4.292 million new cancer cases and 2.814 million deaths in 2015, a large number of clinically confirmed cases. It can effectively prevent the incidence of new cancer and the probability of death by reducing cancer risk factors, as well as reducing it through early screening and effective clinical diagnosis and treatment, saving medical costs, improving prognostic efficacy, and prolonging survival. At present, the latest multimodal medical imaging technologies such as computed tomography (CT), magnetic resonance imaging (MRI) and ultrasound imaging (US) can not only achieve high-resolution imaging of tumor lesions but can also be structured and functionally multimodal Imaging, so as to achieve noninvasive detection of tumor lesions. However, the current clinical imaging-based tumor diagnosis and treatment rely on the doctor's subjective evaluation and operation. However, the current imaging modalities are diversified, coupled with the acquisition of multidimensional spatial data, and the amount of data and information is also increasing. How to pass computer information technology, especially artificial intelligence technology, has always been a research hot spot and difficult point for fully automatic and accurate diagnosis and treatment planning of tumor imaging data. Medical image processing is an important technical means to analyze tumor disease and pathology from multiple dimensions of structure and function, so as to perform diagnosis, treatment planning, and prognosis analysis. Medical image segmentation is a complex and vital step in the field of medical image processing and analysis. Its purpose is to segment normal tissues and organs and tumor lesions in medical images.

With the development of computer information technology and graphic visualization technology, medical diagnosis and treatment are increasingly inseparable from medical imaging. Medical imaging plays an extremely important role in scientific research, teaching, and clinical diagnosis and treatment. At present, the commonly used clinical medical imaging technologies include ultrasound imaging (US), computed tomography (CT), and magnetic resonance imaging (MRI). The increasingly clear and powerful imaging technologies not only realize noninvasive detection of tumor lesions but also serve as an important technical means for monitoring treatment response and prognostic evaluation. In addition, the latest imaging technology can also perform 3D or even 4D dynamic structural and functional imaging, so as to better screen and diagnose and treat diseases. It can provide more abundant key information about tumors and other diseases and, through the latest medical imaging information processing, from extracting potential tumor performance characteristics from the image effectively solves the problem of routine clinical pathological sampling and analysis. MRI has the advantage of high-contrast imaging of soft tissues. At present, it shows very good imaging quality in organs that require high-intensity contrast such as the brain and prostate. However, because the intensity of MRI reconstructed images is not standard, the range of changes is usually large. The subsequent image analysis has brought great challenges. In actual clinical applications, doctors usually combine the performance of tumors and other diseases in different modalities to comprehensively analyze and complete the diagnosis and treatment plan, and everyone agrees that multimodal information can complement each other to eliminate the shortcomings of a single modality and improve the accuracy of image segmentation.

At present, there are many developments in the field of deep learning, but the application in medical imaging is far less extensive than other fields. The following several have their own opinions on medical imaging. Gelfand et al. proposed that if a child-friendly environment is provided for patients and parents, nuclear medicine imaging of children can be best completed and describes a method of minimizing the patient's anxiety and fear. Internationally managed activity guidelines should be used to minimize the radiation dose absorbed by radiopharmaceuticals. The CT exposure parameters may be reduced as the best practice for pediatric diagnostic CT. When CT images are needed only for positioning purposes, the CT exposure parameters may be further reduced. He proposed a method to reduce patient anxiety and fear to improve the diagnostic CT method of pediatrics. Although this method is somewhat effective, the efficiency of this method is too low [1]. Durgadevi and Vijayalakshmi proposed that biomedical image processing has encountered an emotional extension and has become an interdisciplinary research field, with skills derived from interconnected arithmetic, computer science, architecture, insight, material science, science, and drug therapy. PC-assisted instructional processing has become a key part of clinical daily planning. With the new progress of high-tech innovation and the use of different imaging methods, more difficulties have emerged, for example, how to process and decompose a large number of pictures so that first-class data can be provided for disease discovery and treatment. The primary goal of the research is to provide basic ideas and strategies for the preparation of medicinal pictures, and to arouse interest in further inspections and research in restorative imaging processing. Although he applied computer science to medical image processing, it did not bring out the true use of artificial intelligence, and his method was not very convenient [2]. Jeavons proposes equipment and methods for medical diagnosis into images. The device includes an image unit for constructing volume image data by capturing images from tomographic images of a plurality of sample samples, and for constructing an internal three-dimensional image of a diagnostic object of the sample from a viewpoint; a display for displaying a three-dimensional image; an input unit for the inter-voxel image data boundary between the voxel image data of the volume image data closer to the viewpoint than the diagnosis object and the voxel image data associated with the diagnosis object; input parameters for setting the precut plane at the place; the control unit, which controls the structure of the three-dimensional image composed of the image unit based on the precut plane set via the input unit, wherein the control unit is based on one of the parameters input to the input unit to extract the boundary. Although he proposed the method of medical diagnosis into images, his method cannot be used flexibly. The images of tumor cells are generally more complicated than images of other parts, and it is more difficult to image and cut [3].

The innovation of this article is (1) the use of deep learning algorithms. The deep learning model based on convolutional networks currently not only achieves fully automatic target segmentation in the true sense of image segmentation, but more importantly, it is easy to adapt to large-scale image segmentation and application of scale samples. (2) The existing CV model is improved, and accurate and stable ultrasound segmentation of breast tumors is realized, making the image cutting more accurate. (3) Introducing the boundary indicator operator into the CV model makes the curve closer to the real edge on the target boundary and improves the boundary adsorption capacity of the model.

## 2. Application Method of Artificial Intelligence Nuclear Medicine Automated Images

### 2.1. Deep Learning

Deep learning is a branch of machine learning algorithms. The essence is a multilayer neural network structure. Compared with traditional machine learning algorithms, its principle is to better select and change data features by adding network layers, expressive ability [4]. Each layer of the network performs nonlinear mapping on the input data and then outputs the target probability result, and the parameters in the network need to be optimized and iteratively calculated [5]. The calculation process requires back propagation calculation for each layer of the network to achieve the optimization calculation of the objective function and finally obtain the network model parameters [6]. From the perspective of biological neurology theory, the deep learning model better simulates the principle of the human brain signal transmission mechanism. Each output neuron is a weighted calculation nonlinear transmission leading to a deeper neural node, so as to realize the original data in the network effective circulation [7]. In order to solve the problem of calculating the parameters of the network structure, Hubel and Wiesel proposed a convolutional neural network inspired by the research found that the local sensitive and direction-selected neurons exhibit a receptive field in the cat cerebral cortex to perceive external information. The structure effectively reduces the complexity of the feedback neural network [8]. The convolutional neural network not only simulates the human visual perception process well but also avoids the complicated feature extraction process, and the algorithm is easy to achieve parallel calculation. In addition, the weight sharing method effectively reduces the network complexity [9]. It is precisely because of the advantages of convolutional neural networks in computing efficiency and prediction results that this model has been widely used in medical images. There are many related literature reviews on deep learning in the field of medical image imaging and analysis. Literature analysis can see that convolutional neural networks have become the mainstream computing model in the field of medical image analysis. In addition, it can also be seen that the application of deep learning in medical image analysis is concentrated in 2016, showing explosive growth. In medicine, network learning mainly focuses on the research of image segmentation, tissue and organ detection, and tumor target classification. The mainstream training models of deep learning at this stage include unsupervised self-convolutional coding and deep belief networks, convolutional neural networks, recurrent neural networks, etc. [10, 11].

The grayscale statistical feature mainly describes the grayscale information of the image, and there are mainly three different types of grayscale statistical features:

(1) $$\begin{array}{c} \mathrm{Intensity}1=\frac{\sum_{j=1}^{n}\sum_{i=1}^{m}J\left(j,i\right)}{n*m},\\ \mathrm{Intensity}2=\sqrt{\frac{1}{m-1}\overset{n}{\underset{j=1}{\sum }}\overset{m}{\underset{i=1}{\sum }}{\left(J\left(j,i\right)-Jnm\right)}^{2}},\\ \mathrm{Intensity}3=\left\{\begin{array}{c} y_{\left(m+1/2\right)},\\ \frac{y_{m/2}+y_{m+1/2}}{2}. \end{array}\right. \end{array}$$

The above formulas are the average gray-level difference, the gray standard deviation, and the gray-level median.

The gray-level difference feature can be used to express the relationship between the transition area and the nodule area, and the gray-level mean difference is as follows:

(2) $$\begin{array}{c} \mathrm{Intensity}4=\mathrm{mean}\left(J_{K1}\right)-\mathrm{mean}\left(J_{K2}\right). \end{array}$$

The gray-level variance is as follows:

(3) $$\begin{array}{c} \mathrm{Intensity}5=\frac{{\left(\mathrm{mean}\left(J_{K1}\right)-\mathrm{mean}\left(J_{K1}\right)\right)}^{2}}{\mathrm{var}\left(J_{K1}\right)-\mathrm{var}\left(J_{K1}\right)}, \end{array}$$

in which different *J* represent different images, and the grayscale difference feature includes a total of 6-dimensional features.

(4) $$\begin{array}{c} Q\left(j,i|c,\vartheta \right)=\left\{\left(y,x\right)\in n*m|J\left(y,x\right)=j,J\left(y+dy,x+dx\right)=i\right\},\\ Q_{c}\left(j,i\right)=\frac{Q_{c}\left(j,i\right)}{\sum_{j-0}^{L-1}\sum_{i-0}^{L-1}Q_{c}\left(j,i\right)}, \end{array}$$

in which J(y, x) represents a two-dimensional image, the size of which is *n∗m*, *c* represents a displacement vector, and the meaning of the formula is the probability of the appearance of pixel *i* that is the length of pixel *j* and *c*.

(5) $$\begin{array}{c} \mathrm{Intensity}6=\sum_{j=0}^{L-1}\sum_{i=0}^{L-1}\hat{Q_{c}^{2}}\left(j,i\right),\\ \mathrm{Intensity}7=\sum_{m=0}^{L-1}{\left(j-i\right)}^{2}\left\{\sum_{j=0}^{L-1}\sum_{i=0}^{L-1}\hat{Q_{c}^{2}\left(j,i\right)}\right\},\\ \mathrm{Intensity}8=-\sum_{j=0}^{L-1}\sum_{i=0}^{L-1}\hat{Q_{c}}\left(j,i\right)\log\hat{Q_{c}}\left(j,i\right),\\ \mathrm{Intensity}9=\frac{\sum_{j}\sum_{i}ji\hat{Q\left(j,i\right)-\beta_{x}\beta_{y}}}{\alpha_{x}\alpha_{y}},\\ \mathrm{Intensity}10=\sum_{j=0}^{L-1}\sum_{i=0}^{L-1}\frac{\hat{Q_{c}^{2}}\left(j,i\right)}{1+{\left(j-i\right)}^{2}} \end{array}$$

The abovementioned formulas are texture energy, texture contrast, texture entropy, texture correlation, and texture homogeneity, where *β*_*x*_, *β*_*y*_, *α*_*x*_, *α*_*y*_ are the mean and variance of *Q*_*x*_, *Q*_*y*_, respectively:

(6) $$\begin{array}{c} H\left(y,x,\gamma \right)=\left[\begin{array}{cc} H_{yy}\left(y,x,\gamma \right) & H_{yx}\left(y,x,\gamma \right)\\ H_{yx}\left(y,x,\gamma \right) & H_{xx}\left(y,x,\gamma \right) \end{array}\right],\\ H_{yy}=\frac{\partial^{2}f\left(y,x,\partial \right)}{\partial y^{2}},\\ H_{xx}=\frac{\partial^{2}f\left(y,x,\partial \right)}{\partial x^{2}},\\ H_{yx}=\frac{\partial^{2}f\left(y,x,\partial \right)}{\partial y\;\partial x},\\ DE\;T=\lambda^{4}\left(H_{yy}\left(y,x,\gamma \right)H_{xx}\left(y,x,\gamma \right)-H_{yx}^{2}\left(y,x,\gamma \right)\right)=\mu 1*\mu 2, \end{array}$$

in which *H*_*yy*_, *H*_*xx*_, *H*_*yx*_ represent the second derivatives of the point (y, x) on the image in different directions and *μ*1, *μ*2 are the maximum and minimum eigenvalues of the matrix H, respectively.

### 2.2. Principles of Medical Multimodal Imaging

Medical image processing is the first step to analyze tumor diseases. Medical image segmentation is a complex and vital step in the field of medical image imaging and analysis. Its purpose is to detect and distinguish normal tissues and organs and tumor lesions in medical images. The segmented tumor area analyzes the characteristics of the lesion on the image, provides a reliable basis for clinical diagnosis and prognosis management of tumors, and assists doctors in making more accurate diagnosis, treatment planning, and prognostic efficacy analysis [6, 12]. Although there has been a lot of related research work on tumor segmentation of different lesions and different modal images, because medical images are different from natural visual images, they have the complexity of imaging and the variability of lesion performance. The accuracy of the segmentation results is still partially influenced by factors such as volumetric effect, gray inhomogeneity, and noise, and the automatic segmentation of multimodal tumor images is still a complex and challenging task [13, 14]. With the development and maturity of computer information technology and graphic visualization technology, medical diagnosis and treatment are increasingly inseparable from medical imaging. Medical imaging plays an extremely important role in scientific research, teaching, and clinical diagnosis and treatment [15]. Currently commonly used clinical medical imaging technologies include ultrasound imaging (US), computed tomography (CT), and magnetic resonance imaging (MRI). The increasingly clear and powerful imaging technologies not only realize noninvasive detection of tumor lesions but also serve as an important technical means for monitoring treatment response and prognostic evaluation [16]. Ultrasound imaging has been widely used clinically because of its fast imaging speed, no radiation, and low cost, especially for early screening and intraoperative guidance of thyroid, breast, and other parts. However, ultrasound imaging has low signal to noise. Problems such as ratio, image resolution, and imaging depth are difficult to meet the precise diagnosis and treatment goals of tumors; CT is based on the absorption of X-rays in the human body with different densities of tissues and organs to reconstruct images, good imaging quality, but poor imaging results for soft tissues. Sometimes, it is difficult to distinguish the boundaries between tumors and surrounding tissues and organs on soft tissues like liver [17]. MRI has the advantage of high-contrast imaging of soft tissues. At present, it shows very good imaging quality in organs that require high-intensity contrast such as the brain and prostate. However, because the intensity of MRI reconstructed images is not standard, the range of changes is usually large. The subsequent image analysis has brought great challenges. In actual clinical applications, doctors usually combine the performance of tumors and other diseases in different modalities to comprehensively analyze and complete the diagnosis and treatment plan, and everyone agrees that multimodal information can complement each other to eliminate the shortcomings of a single modality and improve the accuracy of image segmentation [18].

### 2.3. Superpixel Boundary Perception Image Block Extraction

Superpixel clusters domain pixels with similar image information such as color, brightness, or texture into a large area. Its essence is also an unsupervised clustering and segmentation algorithm, which uses the characteristics of superpixels to complete image training blocks. The preprocessing can not only greatly improve the efficiency of network training without loss of image information but also make good use of the context space connection information in the image space domain [19, 20]. Since superpixel calculation is based on the operation of image gray information clustering, due to the volume effect phenomenon of CT images, the area information of the liver boundary is very close, which makes it very difficult to distinguish based on gray information. The number selection is very important for boundary fitting. If the superpixel is too large, it will cause boundary segmentation errors [21]; if the superpixel selection is too small, it is equivalent to the traditional pixel block selection, resulting in a large amount of algorithm calculations and more redundant information. It also reduces the performance of the network model. Therefore, the selection of superpixels is also a very important factor in the research that needs to be considered [22].

### 2.4. Artificial Intelligence Multilevel Self-Learning Strategy

The conventional method uses optimization algorithms to solve the model parameters in the loss function of the above formula, but in the process of training the network, all samples are treated equally to update the model parameter values, and the samples are not selectively classified. If the impact of sample quality issues is considered, it will cause the network model to be easily interfered by poor quality image samples. For example, images with tumor lesions or inflammation will make the prostate structure very complicated. These difficulty coefficient samples make the network fall into the local optimum prematurely and cause the network to fail to train [23]. Self-learning strategies have achieved great success in machine learning at present. There is a hard rating strategy to integrate the rich information of samples, through self-learning and multi-instance learning to complete multitarget detection, and the use of self-learning and active learning strategies. To achieve face recognition, these methods are widely used in traditional machine learning algorithms [24].

## 3. Application Experiment of Artificial Intelligence Nuclear Medicine Automated Images

Breast tumor segmentation is the most basic step for accurate tumor measurement and category analysis. It is used for subsequent tumor feature extraction, morphological analysis, and finally input to the classifier for tumor category identification [25–29]. The accuracy of ultrasound segmentation directly affects the follow-up of quantitative analysis and tumor diagnosis and treatment, but because breast tumor images are limited by ultrasound imaging itself, coupled with factors such as clinician manipulation techniques, breast tumors appear low-contrast and limited resolution on ultrasound images. These speckle noises and artifacts make breast ultrasound segmentation, which is still a challenging problem. In order to solve the above problems, this paper proposes a fully automatic segmentation algorithm framework. The segmentation results show that this segmentation algorithm can obtain very good segmentation results, and the performance of the algorithm is further verified through the classification problem.

### 3.1. Subjects

All data in this experiment were collected from the Third People's Hospital affiliated to Sun Yat-sen University. A total of 61 cases were collected, including 32 noninvasive ductal carcinomas (malignant tumors) and 29 fibrous tumors (benign tumors). All these patients had clinical pathology. The gold standard for diagnosis and the data collected by equipment manufacturers are ALOKA, PHILIPS, TOSHIBA, HITACHI, and ESAOTE. Data of each patient contain 5–10 ultrasound images and corresponding pathology reports. The clinician manually divides the data into pixels: level labeling.

### 3.2. Purpose of the Experiment

First, through modeling and denoising analysis of the ultrasonic noise model, the boundary and definition of the ultrasonic image are enhanced, and then an improved OSTU adaptive threshold algorithm is proposed to realize automatic ROI region detection, and finally on the active contour model Chan-Vese (CV). The boundary indication constraint operator is introduced to finally solve the biggest problem of segmentation boundary detection [30–32].

### 3.3. Experimental Process

It is to first calculate the breast ultrasound gray level *L*, then use the OSTU algorithm to calculate the threshold, then get the image foreground and background, then use OSTU on the background to calculate another threshold again while keeping the background unchanged, and finally use the threshold segmentation of the entire image; so far, the experiment is over. Finally, the algorithm model is applied to clinical data for experimental verification [33].

## 4. Application Analysis of Artificial Intelligence Nuclear Medicine Automated Images

### 4.1. Qualitative Visualization Experiment Results

As shown in Figure 1, the malignant breast tumor image is deashed and binarized, and then the threshold is searched for to determine the final tumor location. But through the image, we can clearly see that although threshold segmentation can roughly distinguish the foreground and the background, there are still many peripheral backgrounds that cannot accurately locate the tumor. Figure 1 is deashing and binarization of malignant breast tumor images.

As shown in Figure 2, this is the deashing and binarization of the image of benign breast tumors. We can still see that there are many peripheral backgrounds, but we use the central window boundary method to determine whether the boundary connection area is the same as the central window. The intersection method effectively solves the problem of tumor location [34–37]. (This method is more accurate than using the traditional Grathesh algorithm to automatically find the appropriate threshold value.)

As shown in Figure 3, it is a comparison between the traditional CV algorithm and the artificial intelligence nuclear medicine image based on deep learning in this article. The cutting effect of the algorithm used in this article is significantly greater than that of the traditional CV algorithm. (Although the CV model can detect the boundary well and maintain continuity, the accuracy of the model depends on the setting of the initial contour. This article is improved on this basis, and the boundary operator is introduced to control the boundary convergence, and the boundary indicator is used. Function can make the contour move toward the boundary, to locate the point on the boundary accurately.)

As shown in Figure 4, it is a comparison between the improved Elawady algorithm and the algorithm in this paper. It can be clearly observed that the algorithm in this paper converges more stably on the boundary. Compared with the traditional Elawady algorithm, there will be no boundary overflow, and the algorithm stays stable at the boundary. On the outline, it shows very good stability.

### 4.2. Quantitative Calculation Indicators

As shown in Table 1, the statistical quantitative index results for benign tumor segmentation can be obtained. The similarity between true positive and Jaccard in tumor segmentation in this paper is generally higher than that of the other two traditional algorithms. The false positive of traditional CV algorithm in tumor segmentation is the highest. Yes, the Elawady algorithm has the highest proportion of false negatives.

As shown in Table 2, from the analysis results of the statistical quantitative indicators of malignant tumor segmentation, it can be concluded that the true positive and Jaccard similarities in tumor segmentation in this paper are still higher than those of the other two traditional algorithms.  Figure 5 is the segmentation performance results for benign tumors.

It can be seen from Figure 5 that the accuracy and sensitivity of the CV-ROEMA algorithm are slightly higher than the other two algorithms, and the negative prediction rate is not much different, while the Elawady algorithm is slightly higher in specificity and negative prediction rate.  Figure 6 is the results of segmentation performance of malignant tumors.

It can be seen from Figure 6 that in malignant tumors, CV-ROEMA is much more sensitive than the other two algorithms and is similar in other aspects.  Table 3 is the *p* value of each performance and Kruskal–Wallis index.

It can be seen from Table 3 that in order to test the performance difference between different algorithms, the Kruskal–Wallis evaluation method is used for measurement. From the *p* value, there are certain differences between different algorithm models, indicating that the algorithm performance has been greatly improved.  Table 4 is the *p* value post hoc analysis of different segmentation algorithms.

As can be seen from Table 4, the algorithm model proposed in this paper is significantly different from other algorithms in pairwise comparison, which is much higher in terms of PPV and NPV.

Finally, the experimental results are quantitatively analyzed and compared by quantitative evaluation indicators of true positive, false positive, false negative, Jaccard similarity and sensitivity, specificity, positive prediction rate, and negative prediction rate. We performed a comparative analysis of statistical quantitative index experiments on benign tumors and malignant tumors. From the perspective of quantitative indicators, the segmentation algorithm of this paper has good segmentation performance, and it performs very well in terms of stability and robustness of segmentation accuracy.

### 4.3. Tumor Classification by Different Segmentation Algorithm Results

It can be seen from Table 5 that the learning parameters of network training are configured, and the performance brought by different parameters, combined with the above-mentioned quantitative directional analysis, can compare the advantages and disadvantages of different algorithms.  Table 6 is the effect of different segmentation algorithm results on tumor classification analysis based on morphological features.

It can be seen from Table 6 that the SVM classification algorithm is used to verify and analyze the different segmentation accuracy results, and the tumor morphology analysis is used to evaluate the final impact of the segmentation results on the tumor classification. Finally, it is obvious that the various performances of the algorithm in this paper are better than other algorithms.

## 5. Conclusion

Multimodal medical image segmentation technology has important uses for different clinical application scenarios. CT is based on the principle of absorption of rays in human tissues and organs. The image is reconstructed by back projection, but it is limited by the performance of the imaging sensor and the radiation dose. The problem of balance with the collected data makes CT images very prone to volume effects, making it difficult to identify the boundary in the overlapping regions of breast tissues and other organs. The respective characteristics of these images bring different problems to the image segmentation algorithm. Therefore, through a comprehensive survey of the applied modal images and tissue part segmentation algorithm models represented by breast ultrasound, the advantages and disadvantages of different algorithm models are comprehensively compared and analyzed. The current main segmentation algorithms are based on traditional segmentation algorithms and depth-based segmentation algorithms. Learning segmentation algorithm and traditional segmentation algorithm are difficult to adapt to different modes and target automatic segmentation; therefore, this paper focuses on the analysis based on the principle of deep learning algorithm and the latest algorithm model. In short, the different types of segmentation algorithm models proposed in this paper are all based on data-driven implementations. In view of the performance and problems of different organizations in different modalities, in-depth problem analysis and information mining are carried out, making full use of clinical and theoretical prior knowledge completes model design and parameter optimization. The related algorithm proposed in the paper not only solves the problem of representative modal image segmentation but also can be easily extended to other image analysis applications.

## Figures and Tables

**Figure 1:** Deashing and binarization of malignant breast tumor images.

**Figure 2:** Image deashing and binarization of benign breast tumors.

**Figure 3:** Image cutting of malignant breast tumor. (a) The original image. (b) Standard CV algorithm. (c) Algorithm.

**Figure 4:** Image cutting of benign breast tumor. (a) Original picture. (b) Elawady algorithm. (c) Algorithm.

**Figure 5:** Segmentation performance results for benign tumors.

**Figure 6:** Results of segmentation performance of malignant tumors.

**Table 1:** Analysis results of statistical and quantitative indicators for segmentation of benign tumors.

Methods	TP (%)	FP (%)	FN (%)	JS (%)
Elawady's method	70.38 ± 18.56	1.60 ± 2.41	29.60 ± 18.56	68.51 ± 17.63
Initial contour + CV	84.91 ± 5.58	8.50 ± 15.17	15.07 ± 5.56	78.11 ± 11.62
Initial contour + CV-ROEWA	87.82 ± 5.41	2.41 ± 2.04	12.12 ± 5.41	85.27 ± 5.21

**Table 2:** Analysis results of statistical and quantitative indicators for segmentation of malignant tumors.

Methods	TP (%)	FP (%)	FN (%)	JS (%)
Elawady's method	53.85 ± 28.57	11.75 ± 33.12	46.12 ± 28.57	47.72 ± 26.64
Initial contour + CV	82.43 ± 5.31	2.27 ± 2.86	17.53 ± 5.31	79.71 ± 4.45
Initial contour + CV-ROEWA	85.50 ± 4.85	2.67 ± 3.10	14.45 ± 4.86	82.62 ± 3.56

**Table 3:** *p* value of each performance and Kruskal–Wallis index.

Measurements	Accuracy	Sensitivity	Specificity	PPV	NPV
P	<0.0001	<0.0001	<0.0001	0.0003	0.0002

**Table 4:** *p* value post hoc analysis of different segmentation algorithms.

Measurements	Accuracy	Sensitivity	Specificity	PPV	NPV
p12	0.0238	<0.0001	<0.0001	0.0005	0.0137
p13	<0.0001	<0.0001	<0.0001	0.0042	0.0002
p23	0.2094	0.0528	0.9134	0.8154	0.4613

**Table 5:** SBBS-CNN network training parameter settings.

Epoch	Learning rate	Decay of moving average	Weight decay
20000	0.1	0.9	0.004
60000	0.01	0.9	0.004
100000	0.001	0.9	0.004

**Table 6:** The effect of different segmentation algorithm results on tumor classification analysis based on morphological features.

Methods	Correct	Accuracy (%)	AUC
Manual segmentation	16	84	0.94
Initial contour + CV	13	70	0.90
Initial contour + CV-ROEWA	18	91	0.95

## Data Availability

The simulation experiment data used to support the findings of this study are available from the corresponding author upon request.
